# Cisatracurium inhibits the growth and induces apoptosis of ovarian cancer cells by promoting lincRNA-p21

**DOI:** 10.1080/21655979.2021.1916271

**Published:** 2021-05-04

**Authors:** Dezhang Zhu, Caifeng Shi, Yanan Jiang, Kongjuan Zhu, Xiangzhen Wang, Wei Feng

**Affiliations:** Department of Anesthesiology, Affiliated Hospital of Qingdao University, Qingdao, Shandong, China

**Keywords:** Cisatracurium, long non-coding RNA p21, ovarian cancer, proliferation, apoptosis

## Abstract

As a common muscle relaxant, cisatracurium has shown good antitumor effect on some tumors. Recent studies reported that cisatracurium could inhibit the progression of colon cancer by upregulating tumor suppressor gene p53. However, its role in ovarian cancer and its regulatory effect on p53 and p53 downstream targeting gene long intergenic noncoding RNA p21 (lincRNA-p21) is still unknown. Quantitative Real-time Polymerase Chain Reaction (qRT-PCR) was used to assess the expression of p53, lincRNA-p21 and miR-181b. Cell viability and proliferation were detected by CCK-8 assay and Edu staining, respectively. Wound-healing and Transwell assays were performed to determine the abilities of cell migration and invasion. Apoptosis was evaluated by TUNEL staining. Luciferase reporter assay was conducted to detect the relationship between lincRNA-p21 and miR-181b. As a result, cisatracurium could increase the expressions of p53 and lincRNA-p21 of ovarian cancer cell line (OVCAR-3) in a dose-dependent manner. In addition, cisatracurium significantly inhibited the proliferation, migration and invasion of OVACR-3 cells, and induced apoptosis. However, these above changes in biological function can be attenuated by lincRNA-p21 knockdown. Next, lincRNA-p21 could directly target miR-181b and negatively regulate its expression by luciferase reporter assay. In conclusion, cisatracurium inhibited the progression of OVCAR-3 cells through upregulation of lincRNA-p21 expression activated by p53 inhibiting miR-181b expression. The experimental results provide a new research idea for the application of cisatracurium in ovarian cancer.

## Introduction

As a kind of gynecological malignant tumor, ovarian cancer (OC) has ranked first in the mortality rate of female reproductive system diseases [1]. According to the latest statistics in 18 years, the survival rate of OC patients with within 5 years is no more than 35%[2]. The lack of high sensitivity and specificity for early diagnosis and long-term effective treatment is the main reason for the high mortality of OC. Therefore, to improve the survival rate of OC patients, the search for new tumor markers and therapeutic targets have always been a hotspot in the field of OC research [3,4].

Cisatracurium is a newly developed non-depolarizing muscle relaxant which has been widely used in clinical anesthesia [5,6]. The relaxation strength of cisatracurium is about 4–5 times higher than that of atracurium, and it has the characteristics of good effect, low toxicity and metabolism independent of liver and kidney function, so it has become the most ideal muscle relaxant [7,8]. Because more and more cancer patients need adjuvant anesthesia, it is more important to have a comprehensive understanding of the role about anesthetics in the progression of various cancers. Previous studies have shown that cisatracurium has a good inhibitory effect on tumor progression. For example, cisatracurium inhibited the occurrence and development of epithelial to mesenchymal transition (EMT) in esophageal squamous cell carcinoma (ESCC) cells [9] and suppressed the proliferation, invasion and migration of gastric cancer cells [10]. However, the role of cisatracurium in OC is still unknown. In addition, recent studies reported that cisatracurium inhibited the proliferation, invasion and migration of colon cancer cells by upregulating p53 [11,12]. P53 is located on the short arm of chromosome 17 and belongs to human tumor suppressor gene, which plays a key role in regulating cell cycle, apoptosis, DNA repair and senescence [13–15]. Notably, it is generally believed that p53 can inhibit the biological process of tumors by targeting lincRNA-p21[16]. Extensive studies indicate that long noncoding RNAs (lncRNAs) participate in the regulation of a variety of tumor progressions. Studies showed that lincRNA-p21 could effectively inhibit ESCC [17], colon cancer [18] and hepatocellular carcinoma (HCC) [19]. Whether cisatracurium could affect the progression of OC by regulating lincRNA-p21 activated by p53 is worthy of further study. In consideration of lincRNA-P21 is a newly discovered lncRNA with the capable of adsorbing miRNA, we also investigated the downstream target gene of lincRNA-p21.

Therefore, this paper aims to explore whether cisatracurium can inhibit miR-181b by activating lincRNA-p21 through p53, so as to suppress the ovarian cancer. We firstly detected the expressions of p53 and lincRNA-P21 in OVCAR-3 cells after the treatment of different doses of cisatracurium. Subsequently, CCK-8, Edu staining, migration and invasion assays were used to analyze the effect of cisatracurium on the biological function of OVCAR-3 cells by regulating lincRNA-P21.

## Materials and methods

### Cell culture

Ovarian cancer cell line (OVCAR-3) were obtained from the American Type Culture Collection (ATCC; Rockville, MD USA). Cells were cultured in Dulbecco’s modified Eagle’s medium (DMEM; Hyclone, Logan, UT, USA) containing 10% fetal bovine serum (FBS; Hyclone) and grown at 37°C, 5% CO_2_, and 80% humidity in an incubator. The cells in logarithmic growth phase were taken for experiment. Cells in logarithmic phase were treated with different concentrations of cisatracurium (10, 20 and 40 μM) and cultured for 24, 48 and 72 h, respectively.

### Cell transfection

The plasmids of Ov-NC, Ov-p53, shRNA-NC, shRNA-p53-1, shRNA-p53-2, sh-LincRNA-p21-1, sh-LincRNA-p21-2, Ov-LINC-P21, miR-NC and miR-181b mimic were constructed by GenePharma (Shanghai, China). When the cells in the logarithmic phase reached to 80% confluence, these above plasmids were transfected into OVCAR-3 cells with liposome 2000 (invitrogen) according to the instructions. The transfection efficiency was detected 24 h by qRT-PCR after transfection.

### qRT-PCR analysis

Cells of each group were collected and total RNA was extracted by Trizol reagent (TaKaRa, Japan). RNA synthesized cDNA using Reverse Transcription kit (BioRad, Hercules, CA). Using cDNA as template, real-time PCR was carried out by ABI PRISM 7900HT (Applied Biosystems). U6 and GAPDH were used as internal references. The reaction conductions as follows: 40 cycles (95°C for 5 min, 95°C for 10 s and 60°C for 20 s), and 95°C for 10 s, 60°C for 10 s, 40°C for 30 s. The mRNA expression level of target gene is calculated by 2^−ΔΔ^CT method.

### CCK-8 assay

Cells of each group were inoculated into 96-well plate at a density of 4 × 10^3^ cells per well, and there were 3 complex holes in each group. After 72 h of routine culture, 10 μl of CCK-8 solution was added to each well and continue cultured for 2 h. The OD value of each well at 450 nm wavelength was detected by a microplate reader (BioTek microplate reader). Cell proliferation ability was expressed by OD value.

### EdU staining assay

Cells were inoculated in 96-well plate at 3 × 10^3^ cells/well. Add 100 μl Edu solution (50 μmol/l) to each well, incubate for 1 h, discard the culture medium, then cells were washed with PBS twice. Next, 100 μl of 4% paraformaldehyde was added, incubated for 30 min at room temperature and add 0.5 ml glycine (2 mg/ml) to each well. Subsequently, cells were incubate in a decolorized shaker for 5 min, and discard the glycine solution. The cells were permeabilized in 0.5% TritonX-100 for 10 min and stained with DAPI. Cells were observed by the fluorescence microscope (Olympus, Japan).

### TUNEL staining assay

Apoptosis was determined by the TUNEL detection apoptosis kit (Millipore, MA, USA). Each cell culture slide was incubated with 50 μl TUNEL reaction mixture at 37°C for 1 h. Then, cells were wash with PBS twice and nuclei were counterstained with DAPI. The results were photographed using the fluorescence microscope (Olympus, Japan). Under the microscope, the nucleus of OVCAR-3 cells was stained brown and considerated to be positive.

### Wound-healing assay

Cells were inoculated into 12-well plate at 5 × 10^3^ cells/well. 2 ml DMEM medium was added to each well and continue cultured for 24 h. The cell scratch were made on the plates using a sterile 200 μl pipette tip and take pictures to record the scratch width. After 24 h of culture, the cells were taken out and the width of scratches was photographed under the inverted microscope. Relative scratch healing ratio (%) = (scratch width after 24 h in each group/initial scratch width in each group)/(scratch width after 24 h in control group/initial scratch width in control group) × 100%.

### Transwell assay

DMEM medium without FBS was used to dilute the Metrigel glue (Sigma) and paved on the upper chamber. 100 μl OVCAR-3 cell suspension (2 x 10^5^ cells/ml) was added to the upper chamber covered with Metrigel glue. At the same time, 500 μl DMEM medium containing 10%FBS was added to the lower chamber and cultured for 24 h. The cells in the upper chamber were then lightly wiped with a sterile cotton swab, fixed by 4% paraformaldehyde, stained with crystal violet, and washed with PBS. Invasion cells were observed and counted through the fluorescence microscope (Olympus, Japan).

### Luciferase reporter assay

According to RNA22 analysis, the binding sites of lincRNA-p21 and miR-181b were predicted. HEK293T cells were inoculated into 96-well plates at the density of 3 × 10^4^ cells per well. 24 h later, the lincRNA-p21 3ʹUTR pmirGLO plasmids (containing mutant p21 3ʹUTR or wild-type p21 3ʹUTR) were constructed and cotransfected with miRNA-NC or miR-181b mimic into HEK293T cells with liposome 2000 (invitrogen). They were labeled as miR-NC + lincRNA-p21 WT group, miR-181b + lincRNA-p21 WT group, miR-NC + lincRNA-p21 mut group and miR-181b + lincRNA-p21 mut group, respectively. 48 h after transfection, luciferase activity was detected using the Dual-Luciferase Assay Kit (Promega).

### Western blot analysis

Total protein was extracted by RIPA lysate and the protein concentration was detected by BCA protein assay kit (Beyotime). Then, protein samples were seperated by 10% SDS-PAGE and transferred to PVDF membrane (Millipore). Add 5% skim milk to block the membrane at room temperature for 2 h. After washing the membranes with TBST, the membranes were incubated with primary antibodies against P53 (1:1000; cat. no. #2527; Cell Signaling Technology Inc., USA), MMP2 (1:1000; cat. no. #40994; Cell Signaling Technology Inc., USA), MMP9 (1:1000; cat. no. #13667; Cell Signaling Technology Inc., USA), TIMP1 (1:1000; cat. no. #8946; Cell Signaling Technology Inc., USA), TIMP2 (1:1000; cat. no. #5738; Cell Signaling Technology Inc., USA), Bcl-2 (1:1000; cat. no. #3498; Cell Signaling Technology Inc., USA), Bax (1:1000; cat. no. #5023; Cell Signaling Technology Inc., USA), Caspase-3 (1:1000; cat. no. #14220), Cleaved-caspase3 (1:1000; cat. no. #9661; Cell Signaling Technology Inc., USA) and GAPDH (1:1000; cat. no. #5174; Cell Signaling Technology Inc., USA) at 4°C overnight. Next, the membranes were incubated with horseradish peroxidase-labeled anti-rabbit IgG at room temperature for 2 h. The membrane was developed by he enhanced chemiluminescence (ECL) detection method (Amersham). The gel imaging system (Bio-Rad) was performed to exposure photography. The gray values of protein bands were analyzed by Image J software.

### Statistical analysis

SPSS 22.0 software (SPSS, Inc.) was used for data analysis. Measurement data were expressed as the mean ± standard deviation (SD). Students t-test was used for comparison between the two groups, and One-way ANOVA followed by Turkey’s was used for comparison between the multiple groups .P < 0.05 was considered statistically significant.

## Results

### Cisatracurium inhibits the viability of OVCAR-3 cells and enhances the expression of p53 and lincRNA-p21 in a dose-dependent manner

We first examined the effects of different concentrations (10, 20 and 40 μM) of cisatracurium on the viability of OVCAR-3 cells. CCK-8 results showed that the viability of OVCAR-3 cells gradually decreased with increasing concentration of cisatracurium and 48 h was chosen for the subsequent study (Figure 1a). In addition, PCR and WB results showed that p53 and lincRNA-p21 were up-regulated in OVCAR-3 cells treated with cisatracurium, and the expressions of p53 and lincRNA-p21 increased gradually with rise of cisatracurium concentration at 48 h (Figure 1b and c). After treated with 20 μm cisatracurium for 48 h, the cell viability decreased to 50% of initial values, thus the cisatracurium concentration and the time of treatment of OVCAE-3 cells was determined to be 20 μm and 48 h. Taken together, cisatracurium could significantly inhibit the viability of OVCAR-3 cells and increase the expressions of p53 and lincRNA-p21 in a dose-dependent manner.

**Figure 1.** Cisatracurium inhibits the viability of OVCAR-3 cells and enhances the expression of p53 and lincRNA-p21 in a dose-dependent manner. (a) OVCAR-3 cells were treated with different doses (10, 20 and 40 μM) of cisatracurium for 24, 48 and 72 h, and cell viability was analyzed by CCK-8 assay. (b) Expression of p53 was determined in the OVCAR-3 cells using WB. (c) Expression of p53 was determined in the OVCAR-3 cells using real-time PCR. **p < 0.01 and ***p < 0.001 vs. Control. n = 3

### Cisatracurium inhibits the proliferation of OVCAR-3 cells by activating lincRNA-p21

p53 expression was upregulated in OVCAR-3 cells transfected with Ov-p53 (Figure 2a). p53 expression was decreased in OVCAR-3 cells transfected with shRNA-p53 and showed lower in shRNA-p53-1 group compared with that in shRNA-p53-2 group (Figure 2b). p53 overexpression induced the lincRNA-p21 expression while downregulation of p53 decreased the lincRNA-p21 expression in OVCAR-3 cells (Figure 2c). Next, we explored the effect of cisatracurium on the proliferation of OVCAR-3 cells by regulating lincRNA-p21. LincRNA-p21 expression in OVCAR-3 cells was decreased by lincRNA-p21 knockdown. As shown in Figure 2d, compared with the 20 μM+sh-NC group, lincRNA-p21 expression in 20 μM+sh-LincRNA-p21-1 group was the lowest. Sh-lincRNA-p21-1 plasmid was used for the follow-up experiments. Then, cell proliferation was detected by CCK-8 assay and Edu staining. Results showed that compared with the control group, cisatracurium significantly decreased the viability of OVCAR-3 cells. However, lincRNA-p21 knockdown could alleviate the damage of OVCAR-3 cell proliferation caused by cisatracurium (Figure 2e and f). These data suggest that downregulation of lincRNA-p21 relieve the inhibitory effect of cisatracurium on the proliferation of OVCAR-3 cells.

**Figure 2.** Cisatracurium inhibits the proliferation of OVCAR-3 cells by activating lincRNA-p21. (a) Overexpressed efficiency of p53 expression was detected by real-time PCR. ***p < 0.001 vs. Control. (b) Knockdown efficiency of p53 expression was detected by real-time PCR. ***p < 0.001 vs. Control. (c) LincRNA-p21 expression in OVCAR-3 cells transfected with Ov-p53 or shRNA-p53 was detected by real-time PCR. ***p < 0.001 vs. Control; ^###^p < 0.001 vs. Ov-NC; ^∆∆∆^p < 0.001 vs. shRNA-NC. (d) Knockdown efficiency of lincRNA-p21 expression was detected by real-time PCR. (e) Cell proliferation was determined by CCK-8 assay. (f) Cell proliferation was determined by Edu staining. ***p < 0.001 vs. Control; ^###^p < 0.001 vs. 20 μM+sh-NC. n = 3

### Cisatracurium inhibits migration and invasion of OVCAR-3 cells by activating lincRNA-p21

In addition to the detection of cell proliferation, we also determined the effect of cisatracurium on the migration and invasion of OVCAR-3 cells for 48 h by regulating lincRNA-p21 using wound-healing and Transwell assays. The cell migration and invasion assay results showed that compared with the control group, cisatracurium significantly inhibited the migration and invasion of OVCAR-3. LincRNA-p21 knockdown alleviated the inhibitory effect of cisatracurium on migration and invasion. (Figure 3a–d). In addition, the expression of tumor metastasis-related proteins was detected by western blot analysis. WB results showed that compared with the control group, cisatracurium significantly decreased the expressions of MMP2 and MMP9, whereas increased the expressions of TIMP1 and TIMP2. LincRNA-p21 knockdown could reverse these above changes (Figure 3e). MMPs are a group of proteases that degrade extracellular matrix (ECM) and their viability is regulated by tissue inhibitors of TIMPs. These results suggest that downregulation of lincRNA-p21 alleviate the inhibitory effect of cisatracurium on the migration and invasion of OVCAR-3 cells.

**Figure 3.** Cisatracurium inhibits migration and invasion of OVCAR-3 cells by activating lincRNA-p21. (a and b) Cell migration was determined by wound-healing assay. (c and d) Cell invasion was determined by Transwell assay. (e) The expression of MMP2, MMP9, TIMP1 and TIMP2 were measured by WB. ***p < 0.001 vs. Control; ^#^p < 0.05, ^##^p < 0.01 and ^###^p < 0.001 vs. 20 μM+sh-NC. n = 3

### Cisatracurium promotes apoptosis of OVCAR-3 cells by activating lincRNA-p21

Tunel staining and western blot assay were used to analyze the effect of cisatracurium on apoptosis of OVCAR-3 cells by regulating lincRNA-p21. TUNEL staining results showed that compared with the control group, cisatracurium significantly increased the number of positive apoptotic cells. LincRNA-p21 knockdown significantly reduced the number of positive apoptotic cells (Figure 4a). In addition, we also detected the expression of apoptotic proteins, the results showed that lincRNA-p21 knockdown significantly inhibited the expression of pro-apoptotic protein (Bcl-2 and Cleaved caspase-3) and enhanced the expression of anti-apoptotic protein Bcl-2 (Figure 4b). In general, downregulation of lincRNA-p21 inhibits the inhibitory effect of cisatracurium on apoptosis in OVCAR-3 cells.

**Figure 4.** Cisatracurium promotes apoptosis of OVCAR-3 cells by activating lincRNA-p21. (a) Cell apoptosis were determined by TUNEL staining. (b) The expression levels of apoptosis-related proteins (Bax, Bcl-2, caspase3 and Cleaved caspase3) were determined by WB. ***p < 0.001 vs. Control; ^###^p < 0.001 vs. 20 μM+sh-NC. n = 3

### Cisatracurium inhibits the expression of miR-181b by activating lincRNA-p21

Previous studies showed that lincRNA-p21 could directly target miR-181b to inhibit pulmonary fibrosis, and miR-181b has been confirmed to be highly expressed in ovarian cancer [20,21]. Thus, we examined the regulatory relationship between lincRNA-p21 and miR-181b in ovarian cancer. p53 overexpression suppressed the miR-181b expression while downregulation of p53 promoted the miR-181b expression in OVCAR-3 cells (Figure 5a). LincRNA-p21 expression was decreased in OVCAR-3 cells transfected with shRNA-LINC-P21 and presented lower in shRNA-LINC-P21-1 group compared with that in shRNA-LINC-P21-2 group (Figure 5b). LincRNA-p21 was highly expressed in OVCAR-3 cells transfected with Ov-LINC-P21 (Figure 5c). Downregulation of lincRNA-p21 promoted the miR-181b expression while upregulation of lincRNA-p21 inhibited the miR-181b expression (Figure 5d). As shown in Figure 5e, compared with the control group, cisatracurium significantly decreased the expression of miR-181b in OVCAR-3 cells, while lincRNA-p21 knockdown could reduce the inhibitory effect of cisatracurium on miR-181b. Then, through the construction of miR-181b mimic to increase the expression of miR-181b in OVCAR-3 cells, PCR results showed that compared with the miR-NC group, the expression of miR-181b in miR-181b mimic group was significantly increased (figure 5f). RNA22 analysis predicted the binding of lincRNA-p21 and miR-181b (Figure 5g). Luciferase reporter assay showed that the luciferase activity in the cells cotransfected with miR-181b mimic and lincRNA-p21 3ʹ-UTR mutant vector was lower than that in the cells cotransfected with miR-NC and lincRNA-p21 3ʹ-UTR mutant vector. When OVCAR-3 cells were transfected with lincRNA-p21 3ʹ-UTR mutant vector, miR-181b mimic had almost no effect on the luciferase activity of lincRNA-p21 (Figure 5h). These results suggest that lincRNA-p21 negatively regulated the expression of miR-181b in OVCAR-3 cells.

**Figure 5.** Cisatracurium inhibits the expression of miR-181b by activating lincRNA-p21. (a) miR-181b expression in OVCAR-3 cells transfected with Ov-p53 or shRNA-p53 was detected by real-time PCR. *p < 0.05 and ***p < 0.001 vs. Control; ^∆^p < 0.05 vs. shRNA-NC. (b) Knockdown efficiency of lincRNA-p21 expression was detected by real-time PCR. ***p < 0.001 vs. Control. (c) Overexpressed efficiency of lincRNA-p21 expression was detected by real-time PCR. ***p < 0.001 vs. Control. (d) miR-181b expression in OVCAR-3 cells transfected with shRNA-LINC-P21 or Ov-LINC-P21 was detected by real-time PCR. ***p < 0.001 vs. Control; ^###^p < 0.001 vs. shRNA-NC; ^∆∆∆^p < 0.001 vs. Ov-NC. (e) Effect of lincRNA-p21 on miR-181b expression was determined by real-time PCR. **p < 0.001 vs. 20 μM+sh-NC. (f) Overexpression efficiency of miR-181b expression was detected by real-time PCR. ^###^p < 0.001 vs. miR-NC. (g) Predicted binding sites for miR-181b in lincRNA-p21. (h) The relationship between lincRNA-p21 and miR-181b was determined by luciferase reporter assay in OVCAR-3 cells. n = 3

## Discussion

In all kinds of cancers which are mainly treated by surgery, doctors placed increasing demands requirements on anesthetics to meet their needs of different oncologic surgery. As a very important adjuvant drug of anesthesia in operation, muscle relaxant not only meets the requirements of muscle relaxation in surgery, but also reduces the adverse effects of long-term deep anesthesia on the body [10,22,23]. Therefore, the rational use of muscle relaxants to achieve the optimal muscle relaxation effect and the minimum adverse reactions is the important content of anesthetic research. However, due to the different types of cancer, the effects of muscle relaxants in different cancer surgery are also different. It is worth noting that, in addition to clinical studies, there is little about the role and mechanism of muscle relaxants in various cancer cells. As an ideal muscle relaxant independent of liver and kidney metabolism, cisatracurium has been safely used in clinical anesthesia, but the research on regulating the occurrence and development of cancer cells has not been clearly understood. Therefore, the purpose of this study was to investigate the regulatory effect and potential mechanism of cisatracurium on ovarian cancer cells.

At present, only a few reports have shown that cisatracurium has an inhibitory effect on cancer cells. In ESCC, cisatracurium significantly inhibited the proliferation, migration and invasion of ESCC and induced apoptosis [9]. In HCC, cisatracurium has a significant inhibitory effect on the proliferation, migration and invasion of gastric cancer cells SGC7901 and BGC823[10]. In lung cancer, cisatracurium also significantly suppressed the proliferation and migration of lung cancer cell A549[24]. None of these above studies have deeply studied the regulatory mechanism of cisatracurium in cancer cells, but it is noteworthy that in colorectal cancer (CRC), Yabasin et al reported that cisatracurium could upregulate the expression of p53 protein and then inhibit the metastasis of CRC cells [11]. P53 protein was first found in SV40-transformed cells. It is a 53 kD protein encoded by the house-keeping gene [25]. It has been confirmed that p53 is a negative regulator of cell growth cycle, which is related to important biological functions including cell cycle regulation, DNA repair, cell differentiation, and apoptosis, and plays an important role in inhibiting the growth of cancer cells [26,27]. One previous study showed that more than 50% of p53-deficient mice suffer from malignant tumors, revealing that p53 has the function of tumor suppression [28]. However, no study has shown the effect of p53 on the proliferation, migration and invasion of ovarian cancer cells. In addition, p53 has been widely believed to be able to positively regulate lincRNA-p21 to inhibit the progression of cancer cells [16]. For example, lincRNA-p21 targeting p53 could reduce the development of head and neck squamous cell carcinoma by inhibiting JAK2/STAT3 pathway [29]. At the same time, more and more studies have revealed that lincRNA-p21 plays a tumor suppressor role in a variety of cancers. In HCC, lincRNA-p21 could promote apoptosis of HCC cell HepG2 by activating endoplasmic reticulum stress [30]. In gastric cancer, lincRNA-p21 overexpression effectively inhibited the migration and proliferation of gastric cancer cell MGC-803, and suppressed epithelial-mesenchymal transition (EMT) [31]. In prostate cancer, lincRNA-p21 inhibited the viability and proliferation of prostate cancer cells DU145 and LNCaP by downregulating PKM2[32]. However, the role of lincRNA-P21 in ovarian cancer cells and whether cisatracurium could activate lincRNA-p21 by regulating p53 to inhibit the proliferation, migration and invasion of ovarian cancer cells have not been studied. In this study, cisatracurium could increase the expression of p53 and lincRNA-p21 in ovarian cancer cell OVCAR-3 in a dose-dependent manner. Compared with the control group, lincRNA-p21 knockdown significantly inhibited the proliferation, migration and invasion of OVCAR-3 cells and induce cell apoptosis. These results suggest that lincRNA-p21 can be used as a tumor suppressor in ovarian cancer and is positively regulated by cisatracurium.

Next, we further studied the downstream-targeting genes of lincRNA-p21. lincRNA-p21 is a kind of long noncoding RNA, which could adsorb and regulate miRNA [33]. It has been found that lincRNA-p21 suppressed hepatic fibrosis by targeting miR-181b[20]. MicroRNAs (miRNAs) are an endogenous short-stranded RNAs, with a length of about 19–24 nt, which play an important regulatory role in individual development, cell differentiation, proliferation, apoptosis and other physiological activities [34,35]. Different miR-181b expression can be detected in many types of cancer, and its expression level is related to drug sensitivity, invasion, metastasis and prognosis. For example, miR-181b can interact with STAT3 to regulate glycolysis in colon cancer cells and affect the growth in the mouse xenograft model of colon cancer [36]. MiR-181b overexpression promotes invasion and metastasis of gastric cancer cells through targeting TIMP-3[37]. The expression of miR-181b was upregulated in lung squamous cell carcinoma, indicating that miR-181b may be a new potential biomarker for initial diagnosis of non-small-cell lung cancer [38]. The most important thing is that miR-181b was upregulated in ovarian cancer tissues and promoted the proliferation, invasion and migration of ovarian cancer cells [21]. Our results demonstrated that cisatracurium could reduce the expression of miR-181b in a dose-dependent manner. Meanwhile, we also predicted the binding sites of lincRNA-p21 and miR-181b through the bioinformatic website and verified the targeting relationship between them by luciferase reporter assay. Based on the above results, cisatracurium could activate lincRNA-p21 through upregualting p53 and then inhibit miR-181b, and eventually suppressed the proliferation, migration and migration of OVCAR-3 cells, and induce apoptosis.

## Conclusions

In summary, our results demonstrated that cisatracurium could upregulate p53 to promote lincRNA-p21, and then inhibit miR-181b, to suppress the proliferation, migration and invasion of OVCAR-3 cells and induce tumor cell apoptosis. These findings can provide more in-depth understanding of the antitumor molecular mechanism of cisatracurium and a new perspective for the clinical anesthetic use of ovarian cancer.

## Data Availability

All data generated or analyzed during this study are included in this published article.
